# The Effect of miR-138 on the Function of Follicular Helper T Cells and the Differentiation of B Cells in Osteosarcoma

**DOI:** 10.1155/2021/2057782

**Published:** 2021-11-23

**Authors:** Zhitao Wang, Jianxiao Liang, Shanyong Jiang, Gang Zhao, Jianshu Lu, Baoen Jiang

**Affiliations:** ^1^Department of Traumatic Orthopaedics, Dongying People's Hospital, Shandong, China; ^2^Department of Radiology, Dongying People's Hospital, Shandong, China

## Abstract

**Objective:**

To explore the effect of miR-138 on the function of follicular helper T (Tfh) cells and the differentiation of B cells in osteosarcoma.

**Methods:**

Clinically collect peripheral blood from osteosarcoma (OS) patients and healthy volunteers (HC), as well as OS tumor tissues (OS tumor) and adjacent tissues with normal histology (normal group). The CD4^+^CXCR5^+^Tfh cells of OS patients were screened and isolated by flow cytometry, and the expression of Tfh cell membrane surface antigens PD-1 and CTLA-4 was detected. In addition, qRT-PCR was used to detect the expression of miR-138 in tissues and Tfh cells, and the correlation relationship between miR-138 and PD-1 and CTLA-4 was analyzed. After interference or overexpression of miR-138 in Tfh cells, coculture with untreated B cells was done, and the levels of IL-10, IL-12, IL-21, and INF-*γ* in Tfh cell culture medium and the levels of IgM, IgG, and IgA in B cell culture medium after coculture were measured by ELISA. Flow cytometry was used to detect the expression of B cell membrane surface antigens CD27 and CD38 after coculture.

**Results:**

The rate of PD-1- and CTLA-4 positive cells in the peripheral blood and tissues of the OS group was significantly increased, the expression of miR-138 was significantly reduced, and the expression of miR-138 was negatively correlated with the expression of PD-1 and CTLA-4. In addition, upregulation of miR-138 can lead to a significant increase in the level of IL-10 in the supernatant of Tfh cells and a significant decrease in the levels of IL-12, IL-21, and INF-*γ*, which in turn leads to increased levels of IgM, IgG, and IgA released by B cells. At the same time, it significantly increases the rate of CD27- and CD38-positive cells and promotes the maturation of B cells. Downregulating miR-138 has the opposite effect.

**Conclusion:**

Downregulating the expression of miR-138 in osteosarcoma can improve the dysfunction of CD4^+^CXCR5^+^Tfh cells and promote the differentiation of B cells.

## 1. Introduction

Osteosarcoma (OS) is an extremely aggressive bone malignant tumor originating from the carcinogenesis of mesenchymal stem cells [1]. Its occurrence and development are related to stromal cells, immune infiltration, and a very complex tumor microenvironment [2, 3]. OS is an uncommon tumor. The main affected subjects are children and young adults, accounting for 3-5% of newly diagnosed childhood cancers [4], which tend to occur in the distal femur and proximal tibia [5]. Among them, in patients with tumors, the metastasis to the lungs is greater than 85% [6]. The current clinical treatment for OS includes three aspects: preoperative chemotherapy, surgical resection, and postoperative chemotherapy [5]. Current treatments have significantly improved the prognosis of patients with local OS, but the recurrence rate is as high as 35% [7], and this method is not suitable for patients with advanced, metastatic, or recurrent OS. The prognosis of these types of patients is still very poor [8]. Studies have reported that the survival rate of patients with recurrent OS after two surgical treatments and chemotherapy is 65% of those with local OS, while the survival rate of patients with metastatic OS is less than 20% [5]. The most helpless fact is that adjuvant chemotherapy does not improve the effects of patients with OS lung metastases [9]. Therefore, there is an urgent need to discover new treatment strategies for OS.

Some evidence suggests that OS may be sensitive to immunotherapy. The percentage of CD8^+^ infiltrating lymphocytes in OS tumors is higher than that of other sarcoma subtype 2. The degree of invasion is positively correlated with survival, with OS having a high degree of genomic instability [10]. Follicular helper T cells (Tfh) are a type of CD4^+^ T cells that can help B cells migrate to lymphoid organs to generate and undergo central differentiation into plasma cells in the lymphoid follicles. They can secrete RF, ACPA, and other autoreactive antibodies [11]. Tfh cells are differentiated from BCL-6-induced T cells to express cell membrane-specific antigens. Antigens include CD40 ligand, chemokine receptor 5 (CXCR5), and programmed cell death protein 1 (PD-1) [12, 13]. In addition, Tfh cells can secrete a large number of interleukin-21 (IL-21), IL-6, IL-10, and INF-*γ* and other cytokines and promote the secretion of immune factors such as IgM, IgG, and IgA from B cells and promote the maturation of B cells [14]. Studies have shown that Tfh cells are the key cells of the body's immune response and can promote the growth and differentiation of B lymphocytes [15]. After B cells mature, immune responses can occur to eliminate pathogens. Studies have pointed out that in patients with OS, the cytokine secretion capacity and cell proliferation capacity of Tfh cells are significantly reduced, which may be why the body cannot counteract the development of OS [16]. However, there is no research on the mechanism of Tfh cell damage in OS.

MicroRNAs (miRNAs) are small, noncoding RNAs with a size of about 22 nt, and it has been confirmed that miRNA is involved in the occurrence and development of tumor cells and the exchange of information with the external microenvironment [17, 18]. Gong et al. found that metastatic OS cells can secrete exosomes with miR-675, transmit signals to stromal cells, reduce the expression of their CANN1 gene, and promote tumor cell migration and invasion [16]. Liu et al. found that OS cells can promote the expression of the IL-6R gene by reducing the transmission of miR-451 signals to vascular epithelial cells and enhance their angiogenesis ability [19]. Studies have shown that miR-138-5p can be used as a biomarker for the poor prognosis of OS in children, adolescents, and young adults [20]. And miR-138 can directly target TNFAIP8 and play a tumor suppressor effect in OS [21]. Moreover, miR-138 inhibits tumors and enhances cisplatin-induced apoptosis in OS cells by targeting EZH2 [22]. These studies confirm the involvement of miR-138 in inhibiting the progression of OS. However, there are few studies on whether miR-138 affects Tfh cells in OS. Therefore, this paper detects the expression of miR-138 related to OS, reveals its influence on Tfh cell function, and proposes new ideas for the treatment of OS.

## 2. Materials and Methods

### 2.1. Tissue Specimens

30 cases of OS patients who were diagnosed and treated in our hospital and 30 healthy volunteers (HC) who underwent physical examinations in our hospital during the same period were collected. The peripheral blood of the two groups of patients was collected, as well as the tumor tissues of patients with OS (OS tumor) and adjacent tissues with normal histology (normal). All patients in this study gave informed consent to the study and signed an informed consent form. This study was approved by the Clinical Trial Ethics Committee of Dongying People's Hospital and strictly followed the *Declaration of Helsinki*.

### 2.2. Separation and Detection of Tfh Cells in Blood and Tissues

Peripheral blood of patients in the HC group and OS group was collected, and lymphocyte separation solution (Solarbio, USA) was added. The single-cell suspension was collected after 30 min at 4°C 900 r/min. The tumor tissues and adjacent tissues of patients with OS were ground using a sieve, the single-cell suspension was collected, the supernatant was discarded after centrifugation at 500 g at 4°C for 5 min, and the cell pellet was collected. 40 *μ*l magnetic-activated cell sorting (MACS) buffer was used for resuspension with the addition of 10 *μ*l CD4^+^ T cell Biotin-Antibody Cocktail, incubated at 4°C in the dark for 5 min. 1 ml MACS buffer was then added to wash and centrifuged at 1500 r/min for 5 min before discarding the supernatant. After resuspending the cells in 30 *μ*l MACS buffer, 20 *μ*l CD4^+^ T cell Microbead Cocktail was added, incubated at 4°C in the dark for 10 min before adding 1 ml MACS buffer to wash, and centrifuged at 1,500 r/min for 5 min, and the supernatant was discarded. After that, the sorting column-MS column, magnet block, and magnetic stand were placed, the column was moistened with 500 *μ*l MACS buffer, and the cells were resuspended in 500 *μ*l MACS buffer. The cell suspension was passed through the column, collect the effluent and wash the column with 500 *μ*l MACS buffer 3 times, and collect the effluent. Collect the cell suspension obtained 4 times, centrifuge at 1500 r/min for 5 min, and discard the supernatant, and the obtained cells are CD4^+^ T cells. After adding 2 ml of PBS buffer, the supernatant was collected by centrifugation at 1500 rpm for 5 min, transferred into a flow tube, added with CXCR5, PD-1, and CTLA-4 fluorescent antibodies (BD, USA), and mixed well. After incubation at room temperature for 30 min, the cells were washed with PBS and Tfh cells were detected by flow cytometry [23]. The collection solution was PBS containing 30% FCS, and the cells in the collection fluid were cultured in an incubator.

### 2.3. B Cell Isolation

The peripheral blood of patients in the HC and OS groups was collected, lymphocyte separation solution (Solarbio, USA) was added, and single-cell suspension was collected after 30 min at 4°C 900 r/min. A CD19 antibody was used to label B cells. Every 10^7^ cells were resuspended with 90 *μ*l of MACS buffer, added with 10 *μ*l of anti-CD19 microbeads after mixing, mixed well by tapping the bottom of the tube, and incubated at 4°C for 15 min in the dark. 1 ml buffer was added to rinse the cells and centrifuged at 300 g for 10 min, and the supernatant was discarded before adding 1 ml buffer to resuspend the cells. The MidiMACS sorter was used to sort and collect CD19^+^ B cells.

### 2.4. Tfh Cell Transfection

Tfh cells isolated from the peripheral blood of OS patients were seeded in a 6-well plate at 2 × 10^5^ cells/well. When the growth and confluence reached 60-70%, the lipo 2000 kit (Thermo Fisher, USA) was used to transfect NC mimics, miR-138 mimics, NC inhibitor, and miR-138 inhibitor. After 6 h of transfection, the culture medium was replaced with a fresh medium and cultured for 48 hours.

### 2.5. Cocultivation of Tfh Cells and B Cells

Untreated B cells (3 × 10^4^ cells/well) and transfected Tfh cells (3 × 10^4^ cells/well) were placed and cultured in AIM-V medium (Life Technologies) with *Staphylococcal enterotoxin* B (SEB, 100 ng/ml, Toxin Technology). After 7 days, the levels of IgM, IgG, and IgA in the B cell culture supernatant were determined [24].

### 2.6. qRT-PCR

The total RNA of cells is extracted by the method of TRizol. cDNA was prepared according to the random primer reverse transcription kit (Thermo, USA). The expression level of each mRNA was detected according to the instructions of the SYBR GREEN kit (TaKaRa, Japan), with GAPDH and U6 used as internal controls, and the experiment was set to 6 replicates. The experimental data obtained by qRT-PCR was calculated using the 2^−ΔΔCt^ method to calculate the relative expression of the target gene. The primer sequence is shown in Table 1.

### 2.7. ELISA

After the transfected Tfh cells were cultured for 2 days, the culture supernatant of each cell group was collected and centrifuged at 4°C and 1000 r/min for 5 min to remove cell debris, and the supernatant was transferred to a new sterile centrifuge tube. The levels of cytokines IL-10, IL-12, IL-21, and INF-*γ* in the culture supernatant were detected according to the ELISA reagent instructions (Nanjing Jianshe, China).

### 2.8. Statistical Analysis

Statistical analysis was performed using SPSS 26.0. The comparison between the two groups was analyzed by an independent sample *t*-test, and the comparison between multiple groups was analyzed by a one-way analysis of variance. The results were expressed as mean ± standard deviation (SD). The correlation between miR-138 and PD-1 expression in peripheral blood was analyzed by the Pearson correlation. *p* < 0.05 was used as the criterion for judging the significance of the difference.

## 3. Results

### 3.1. Tfh Cells Were Increased in Peripheral Blood and Tumor Tissues of Patients with Osteosarcoma

Firstly, Tfh cells in peripheral blood and tumor tissues of OS patients were screened by flow cytometry. Flow cytometry (Figures 1(a) and 1(b)) showed that compared with the HC group, the proportion of CD4^+^CXCR5^+^Tfh cells in the peripheral blood and tumor tissue of OS patients was significantly increased. Further detection of CD4^+^CXCR5^+^Tfh cell surface-related antigen PD-1 and CTLA-4 expression found that the expression of PD-1 and CTLA-4 in peripheral blood and tissues of OS patients was significantly increased (Figures 1(c) and 1(d)).

### 3.2. miR-138 Is Underexpressed in Osteosarcoma Patients

The expression of miR-138 in OS and its association with Tfh cells was further examined. The results showed that the expression level of miR-138 in the peripheral blood of patients in the OS group was significantly lower than that of the HC group (Figure 2(a)). At the same time, the correlation analysis revealed that miR-138 was negatively correlated with the expression of PD-1 and CTLA-4 (Figures 2(b) and 2(c)). In addition, the expression level of miR-138 was also significantly downregulated in tumor tissues of OS patients compared with normal adjacent tissues, and it was negatively correlated with the expression of PD-1 and CTLA-4 (Figures 2(d)–2(f)). These results suggest that there may be an effect between miR-138 and Tfh cells, which in turn acts on the development of OS.

### 3.3. Upregulation of miR-138 Expression Can Promote the Immune Function of Tfh Cells and the Differentiation of B Cells

Studies have shown that T cells can increase the affinity of B cells, thereby inducing the maturation of B cells. Mature B cells can produce a diverse B cell pool and high-affinity B cell antigen receptors (BCRs) for pathogen clearance [25]. Therefore, we further studied the effect of miR-138 expression on the maturation of OS Tfh cells and B cells. We transfected miR-138 mimics and their control mimic NC in the peripheral blood of OS patients. The qRT-PCR results showed that compared with the mi-NC group, the expression of miR-138 in the Tfh cells of the miR-138 mimic group was significantly increased, confirming successful transfection (Figure 3(a)). The levels of IL-10, IL-12, IL-21, and INF-*γ* released by Tfh cells were further tested, and it was found that the levels of IL-10 were significantly reduced while IL-12, IL-21, and INF-*γ* significantly increased in Tfh cells of OS patients. After overexpression of miR-138, IL-10 levels increased compared with the mi-NC/OS group, while IL-12, IL-21, and INF-*γ* levels were significantly decreased (Figures 3(b)–3(e)). Subsequently, Tfh cells were cocultured with untreated B cells to detect the effect of miR-138 on B cell maturation. The results found that the levels of IgM, IgG, and IgA released by B cells in OS patients were significantly reduced, and the levels of B cell maturation markers CD27 and CD38 were significantly reduced. After overexpression of miR-138, Tfh cells would promote an increase in IgM, IgG, and IgA levels released from B cells (Figures 3(f)–3(h)). At the same time, the levels of CD27 and CD38 were significantly upregulated compared with the mi-NC/OS group (Figure 3(i)). After interfering with the expression of miR-138, the above results all showed the opposite trend (Figures 4(a)–4(i)). This shows that miR-138 can affect the immune function of Tfh cells, which in turn affects the maturation of B cells.

## 4. Discussion

The body's immune disorder is a key factor in accelerating the development of OS [26]. It has been reported that the content of CD4^+^CXCR5^+^Tfh cells in the peripheral blood of OS patients is increased [27], and Tfh cells can induce B cell activation and produce various cytokines [28], suggesting that Tfh cells play a key role in the occurrence of OS. However, studies have shown that the increase in Tfh cells cannot increase the level of IL-21 in the peripheral blood of patients [29], which indicates that there may be other regulatory pathways in OS to limit the body to compensate for functional damage by increasing the number of Tfh cells. Helping B cells to react with antibodies is the main function of CD4^+^ T cells [30], and Tfh cells are essential for the activation of B cells [28]. B cell maturation plays an important role in the elimination of pathogens. Studies have shown that cytokine signaling is essential for cell survival, proliferation, differentiation, and undergoing programmed cell death. Studies have pointed out that IL-12, IL-21, and INF-*γ* can promote Tfh cell differentiation efficiency [31], while IL-21 and INF-*γ* can stimulate CD4^+^ T cells to express CXCR5 through the STAT3 signaling pathway [32], and IL-12 can function indirectly by stimulating IL-21 [33]. However, the STAT3 signaling pathway will also activate the expression of PD-1 to inhibit ICOS signaling, thereby reducing its function of promoting B cell differentiation [34]. The experimental results of this study showed that Tfh cells increased significantly in the peripheral blood and tumor tissues of OS patients, but the level of IL-10 released by Tfh cells of OS group patients was significantly reduced in the HC group while IL-12, IL-21, and INF-*γ* levels have risen significantly. After cocultivation of Tfh cells and B cells in the OS group, the levels of IgM, IgG, and IgA released by B cells were significantly lower than those in the HC group. It is suggested that although the number of Tfh cells in OS patients increases, the function of Tfh cells and the maturation of B cells can be significantly inhibited by various cytokines.

At the same time, numerous studies have confirmed that miRNA is an efficient signal transmission carrier; miR-138 has been proven to regulate many biological processes, including embryonic morphogenesis and development related to stem cell differentiation [35]. And some studies have shown that miR-138 can target and regulate the expression of cytotoxic T lymphocyte-associated molecule-4 (CTLA-4) and programmed cell death ligand-1 (PD-1) genes, thereby playing a role in regulating the body's immunity function [36]. Among them, CTLA-4 and PD-1 are negative regulators of T cell activation, promoting T cell apoptosis and mediating tumor immunosuppression by inducing the expression of T cell suppressor factor (Treg) [37, 38]. Therefore, this study took miR-138 as the research object and found that the expression of miR-138 in the peripheral blood and tumor tissues of patients with OS was significantly reduced, and it was negatively correlated with the expression of CTLA-4 and PD-1. This suggests that miR-138 may be a signal molecule for OS to regulate the tumor microenvironment.

In a variety of cancers, the expression of miR-138 is downregulated, and miR-138 has been shown to have tumor suppressor effects [39]. The current study reveals that miR-138 has the ability to interact with the immune system. Li et al. found that miR-138 inhibits the occurrence and development of oral squamous cell carcinoma (OSCC) by immunostimulating T cells [40]. Fu et al. [41] pointed out that miR-138 can inhibit the occurrence and development of psoriasis by targeting runt-related transcription factor 3 (RUNX3) and regulating the Th1/Th2 ratio in CD4^+^ T cells. In order to verify the effect of miR-138 on the immune environment in OS, this experiment observed its impact on Tfh cell function and B cell maturation after interfering or overexpressing miR-138 expression in Tfh cells. The results showed that the upregulation of miR-138 can significantly reduce the levels of IL-12, IL-21, and INF-*γ* in Tfh cells but increase the level of the anti-inflammatory factor IL-10 and promote the increase in immune factor IgM, IgG, and IgA contents in B cells during coculture. But the effect after interference with miR-138 was the opposite. It shows that the increased expression of miR-138 can significantly improve the immune function of Tfh cells and the differentiation of B cells. It can be seen that OS may inhibit the function of Tfh cells by reducing the expression of miR-138, thereby inhibiting the maturation of B cells, which in turn affects the body's immune response.

## 5. Conclusion

In summary, OS may inhibit the immune function of Tfh cells and B cell differentiation by reducing the expression of miR-138, leading to a significant reduction in the levels of IL-10, IgM, IgG, and IgA and the rate of CD27- and CD38-positive cells, as well as increasing the levels of IL-12, IL-21, and INF-*γ* to promote the occurrence and development of OS. These results suggest that miR-138 can be used as a potential biomarker and a new therapeutic target of OS. However, this study failed to fully clarify the process of how miR-138 exerts its biological functions. Therefore, further *in vivo* experimental studies are needed to better reveal the mechanism of immune disorders caused by OS and to provide an effective theoretical basis for the treatment of the disease.

## Figures and Tables

**Figure 1:** The content of Tfh cells in peripheral blood and tumor tissues of patients with osteosarcoma. (a) Flow cytometry was used to detect CD4^+^CXCR5^+^Tfh cell content in peripheral blood of patients in the HC group and OS group. (b) Flow cytometry was used to detect CD4^+^CXCR5^+^Tfh cell content in tissues of the OS group. (c) Flow cytometry was used to detect the expression of PD-1 and CTLA-4 in CD4^+^CXCR5^+^Tfh cells in the peripheral blood of patients in the HC group and OS group (^∗∗^*p* < 0.01*vs.* HC group). (d) Flow cytometry was used to detect the expression of PD-1 and CTLA-4 in CD4^+^CXCR5^+^Tfh cells in the tissues of patients in the OS group (^∗∗^*p* < 0.01*vs.* normal group).

**Figure 2:** The expression of miR-138 in peripheral blood and tumor tissues of patients with osteosarcoma. (a) qRT-PCR was used to detect the expression of miR-138 in the peripheral blood of patients in the HC and OS groups (^∗∗^*p* < 0.01*vs.* HC group). (b) Pearson correlation was used to analyze the correlation between the expression of miR-138 and PD-1 in the peripheral blood of OS patients. (c) Pearson correlation was used to analyze the correlation between the expression of miR-138 and CTLA-4 in the peripheral blood of OS patients. (d) qRT-PCR was used to detect the expression of miR-138 in cancer tissues and adjacent tissues of OS patients (^∗∗^*p* < 0.01*vs.* normal group). (e) Pearson correlation was used to analyze the correlation between the expression of miR-138 and PD-1 in the cancer tissue of patients with osteosarcoma. (f) Pearson correlation was used to analyze the correlation between the expression of miR-138 and CTLA-4 in the cancer tissue of patients with osteosarcoma.

**Figure 3:** The effect of upregulation of miR-138 expression on the immune function and B cell differentiation of osteosarcoma Tfh cells. After Tfh cells were transfected with miR-138 mimics (miR-138) and its control mimic NC (mi-NC), (a) qRT-PCR was used to detect the expression of miR-138 in Tfh cells. (b–e) ELISA was used to detect IL-12 (b), IL-21 (c), INF-*γ* (d), and IL-10 (e) expression in the supernatant of Tfh cells. (f–h) Tfh cells were cocultured with B cells, and ELISA was used to detect the expression of IgM (f), IgG (g), and IgA (h) in the supernatant of each group of cells. (i) After Tfh cells were cocultured with B cells, the rate of CD27- and CD38-positive cells in B cells was detected by flow cytometry. ^∗∗^*p* < 0.01*vs.* HC group, ^##^*p* < 0.01*vs.* mi-NC/OS group.

**Figure 4:** The effect of upregulation of miR-138 expression on the immune function of osteosarcoma Tfh cells and the differentiation of B cells. After Tfh cells were transfected with the miR-138 inhibitor (in-miR-138) and its control inhibitor NC (in-NC), (a) qRT-PCR was used to detect the expression of miR-138 in Tfh cells. (b–e) ELISA was used to detect the expression of IL-12 (b), IL-21 (c), INF-*γ* (d), and IL-10 (e) in the supernatant of Tfh cells. (f–h) Tfh cells were cocultured with B cells, and the expression of IgM (f), IgG (g), and IgA (h) in the supernatant of each group of cells was detected by ELISA. (i) After Tfh cells were cocultured with B cells, the rate of CD27- and CD38-positive cells in B cells was detected by flow cytometry. ^∗∗^*p* < 0.01*vs.* HC group, ^##^*p* < 0.01*vs.* in-NC/OS group.

**Table 1:** Primer sequence.

RNA	Sequences (5′ to 3′)
miR-138	F: GCTGGTGTTGTGAATCAG
	R: GAACATGTCTGCGTATCTC
PD-1	F: AAGGCGCAGATCAAAGAGAGCC
	R: CAACCACCAGGGTTTGGAACTG
CTLA-4	F: ACGGGACTCTACATCTGCAAGG
	R: GGAGGAAGTCAGAATCTGGGCA
U6	F: CTCGCTTCGGCAGCACAT
	R: TTTGCGTGTCATCCTTGCG
GAPDH	F: CATCACTGCCACCCAGAAGACTG
	R: ATGCCAGTGAGCTTCCCGTTCAG

## Data Availability

The data used to support the findings of this study are available from the corresponding author upon request.
